# A Molecular Mechanism Study to Reveal Hirudin's Downregulation to PI3K/AKT Signaling Pathway through Decreasing PDGFR*β* in Renal Fibrosis Treatment

This article has been retracted.

**DOI:** 10.1155/2022/5481552

**Published:** 2022-09-07

**Authors:** Ying Li, Ling Zhang, Weijian Xiong, Xuan Gao, Yanying Xiong, Wei Sun

**Affiliations:** ^1^Nanjing University of Chinese Medicine, Nanjing 210023, China; ^2^Department of Nephrology, Chongqing Hospital of Traditional Chinese Medicine, Chongqing 400021, China; ^3^Department of Nephrology, Jiangsu Province Hospital of Chinese Medicine (Affiliated Hospital of Nanjing University of Chinese Medicine), 210029, China

## Abstract

Chronic kidney disease (CKD) is identified as a widespread chronic progressive disease jeopardizing public health which characterized by gradually loss of renal function. However, there is no efficient therapy to prevail over this disease. Our study was attempting to reveal hirudin's regulation to renal fibrosis as well as the molecular mechanism. We built renal fibrosis models on both cell and animal levels, which were subsequently given with hirudin disposal; then, we performed the transwell assay to estimate the cells' migration and had our detection to relevant proteins with western blot and immunofluorescence. Finally, we commenced both the identification and the determination to the hirudin targeted proteins and its downstream signaling pathways with the methods of network pharmacology. And the results turned out that when it was compared with the model group, the group with hirudin addition came with the suppression in the migration of renal tubular epithelial cells NRK-52E and with a conspicuous decline in the expressions of fibronectin, N-cadherin, vimentin, TGF-*β*, and snail. After that, we predicted that there were 17 hirudin target points mainly involving in the PI3K-AKT signaling pathway. Our outcomes of the animal level demonstrated that the conditions of interstitial fibrosis, severe tubular dilatation or atrophy, inflammatory cell infiltration, and massive accumulation of interstitial collagen in the model group were withdrawn after the addition of hirudin. In addition, p-PDGFR*β*, p-PI3K, and p-AKT protein expressions were significantly reduced, and the PI3K/AKT pathway was downregulated after hirudin treatment in the model group of NRK-52E cells and animals. Therefore, we had our conclusion that hirudin is capable of suppressing the PI3K-AKT signaling pathway as well as the EMT by decreasing PDGFR*β* phosphorylation.

## 1. Introduction

The increasing number of chronic kidney disease (CKD) patients has become a prevalent common health matter worldwide and is a major disease driving death globally. Pathologically speaking, CKD is the major cause of progressive and irreversible renal tissue damage, renal dysfunction, and nephron loss [1]. Renal fibrosis is the most important trait of CKD and a common progression for many categories of CKD into end-stage renal disease (ESRD) as well [2]. Manifestations of renal fibrosis are primarily the accumulation of extracellular matrix (ECM), inflammatory response, epithelial-to-mesenchymal transition (EMT), and the activation and the proliferation of fibroblasts [3]. Growing evidence has proved that the EMT is the crucial cause for the occurrence and the development of renal interstitial fibrosis (RIF) [4].

EMT refers to the transition of renal tubular epithelial cells' phenotype, which proves to be the reduced expression of epithelial markers like E-cadherin. Furthermore, the contents of mesenchymal markers such as *α*-smooth muscle actin (*α*-SMA) and vimentin are increased [5, 6]. EMT and ECM depositions are separately deemed to be the most important and the most common features within renal fibrosis course. They are also the reasons for the occurrence and the development in RIF [3, 7].

PI3K/AKT is a typical signaling pathway covering the aspects including cell growth, apoptosis, metastasis, and drug resistance manipulations [8]. Recent studies show that the PI3K/AKT axis is also essential in EMT regulation [9, 10]. The series of cytokines including fibroblast growth factor transforming growth factor-*β* (TGF-*β*), platelet-derived growth factor (PDGF), and tumor necrosis factor-*α* (TNF-*α*) are required in EMT activation [9]. Vascular endothelial growth factor family member, the PDGF, broadly speaking, is made of the homologous or the heterodimer molecules of A, B, C, and D polypeptide chains bonded with disulfide linkages; categorized with the components, there are 5 subtypes of the PDGF molecules (PDGF-AA, BB, AB, CC, and DD) [11]. Those PDGF molecules function as the major regulators in cellular proliferation and migration, inflammation, tissue permeability, and involvement in extracellular matrix deposition and so on [11, 12]. PDGFR is the receptor of PDGF molecules, which is phosphorylated and then combined with the p85 subunit of the phosphoinositide 3-kinase (PI3K) in renal fibrosis course via SH2 domain structure so that the downstream molecules in the AKT pathway are to be activated [13].

Hirudin is the main active compound in leech extract. Its anticoagulant and antithrombotic properties provide more molecular targets for disease treatment, clinical research, and drug synthesis, and its application prospect is inconceivable [14]. Hirudin is a small protein (polypeptide) composed of 65~66 amino acid residues weighing around 7000 Da [15]. The disulfide bonds in hirudin determine the stability of its tertiary structure. The natural hirudin molecule has 5 amino acid hydrophobic groups at the N-terminus, and a hydrophilic group enriched in acidic amino acid residues is found at the C-terminus. There have been many reports confirming the effectiveness of hirudin in treating kidney diseases. Xie et al. reported the efficacy of hirudin in improving RIF in unilateral ureteral obstruction (UUO) mice, and Han et al. have demonstrated that hirudin protects against kidney damage by inhibiting inflammation via the P38 MAPK/NF-*κ*B pathway [16, 17]. Moreover, the study verified that hirudin ameliorates RIF via regulating TGF-*β* /Smad and NF-*κ*B signaling in UUO rat model [18] and the further study proved that hirudin can reduce related markers' expression of ECM via the HIF-1*α*/VEGF signaling pathway in diabetic kidney disease rats [19].

The inhibitory efficacy of hirudin on EMT is proved in this study; that is, hirudin hinders the PI3K/AKT signaling pathway, thereby inhibiting EMT and ultimately alleviating the process of renal fibrosis.

## 2. Material and Methods

### 2.1. Cell Cultures

NRK-52E is utilized for the rat tubular epithelial cell line (a layer of cells on the outside of the kidney tubules) and is acquired from American Type Culture Collection (ATCC) and then is cultivated with the DMEM (Gibco, Carlsbad, CA) containing 0.1 mM nonessential amino acids and supplemented with 10% FBS, 100 mg/ml streptomycin, and 100 U/ml penicillin. Then, these cells were placed in a 5% CO_2_, 37°C incubator. These cells were grouped into 3 groups: control (cultured with glucose-free DMEM and with no intervention), model (cultured with 25 mmol/l glucose and intervened with 10 nmol/l AngII), and model+hirudin group (cultured with 25 mmol/l glucose, 10 nmol/l AngII, and 100 *μ*g/ml hirudin). Cells of each group were grown in 3 individual wells and cultured in the condition of 37°C and 5% CO_2_ for 3 days with one medium changed every 24 hours.

### 2.2. Transwell Assay

Transwell assay for the cellular invasion evaluation was performed with Cell Culture Insert (Falcon, USA). Briefly, we rinsed the cells with PBS and then, the resuspension of cells was exerted with 200 ml medium. After that, we had these cells grown in the upper chamber coated with Matrigel (BD Biosciences, USA) and added 10% FBS in the lower chamber. Twenty-four hours after these chambers were kept in the incubator with 5% CO_2_ at 37°C, the fixation of cells was performed using 4% paraformaldehyde (PFA); crystal violet was utilized for staining for 3 min, then determined under Axio Imager A2 (ZEISS, Germany).

### 2.3. Western Blots

The extraction of protein lysates containing target protein in kidney tissues was obtained via cell lysis buffer (Beyotime, China) mixed with 1 mM of phenylmethanesulfonyl fluoride (PMSF). Then, centrifugation was carried out at 4°C and 12000 rpm for 20 min; supernatant was collected on the basis of which the protein content was determined. The retrieval of membrane and cytoplasmic proteins using Membrane and Cytosol Protein Extraction Kit (# P0033; Beyotime) for was performed. Proteins were separated by electrophoresis by employing 10% SDS/PAGE at 80 V and then transferred to PDVF membranes (Millipore, Billerica, MA) lasting for 2 h at 60 V and a constant current of 250 mA. Subsequently, the PDVF membrane was successively operated through blocking with 5% skim milk, washing with TBST, and incubation with primary antibody. The immunoblots of detected proteins were probed with antibodies. Protein immunoblots were visualized through exposure by exploiting Ultrasensitive chemiluminescence substrate kits acquired from New Cell & Molecular Biotech Co, Ltd.

### 2.4. qPCR

The RNA was retrieved using RNAiso Plus (9108; Takara), and concentration was determined via detecting OD value (NanoDrop One/One C; Thermo). The DNA synthesis was then performed by reverse transcription according to the PrimeScript RT reagent Kit (Takara). 2 × T5 Fast qPCR Mix (SYBR Green I) provided by Tsingke Biotechnology Co., Ltd. was employed to conduct the qPCR experiment with primers as follows: fibronectin-F: 5′-TGGTTTGGTCTGGGATCAAT-3′, fibronectin-R: 5′-ACAGTGCTGCAGGTCAGATG-3′; N-cadherin-F: 5′-GACGGTTCGCCATCCAGAC-3′, N-cadherin-R: 5′-TCGATTGGTTTGACCACGG-3′; vimentin-F: 5′-GCTTCAGAGAGAGGAAGCCGAAAA-3′, vimentin-R: 5′-TTTCCAAGCCGACCTCACGG-3′; TGF-*β*-F: 5′-ACTACTACGCCAAGGAGGTCAC-3′, TGF-*β*-R: 5′-TGCTTGAACTTGTCATAGATTTCG-3′; snail-F: 5′-CTGCGGGAAGGCCTTCTCT-3′, snail-R: 5′-CGCCTGGCACTGGTACTTCTT-3′.

### 2.5. Immunofluorescence

The relative rabbit polyclonal antibodies of fibronectin and N-cadherin were employed for protein probing. The visualization for fluorescence signals of proteins was conducted by using Alexa Fluor 594-conjugated antibody (Invitrogen), and staining of the nucleus was performed using 1 mg/ml DAPI for 3 min. Finally, the analysis of stained sections was conducted by a microscope (Leica TCS SP8, Germany).

### 2.6. Prediction on Hirudin Target Proteins, the PPI Network Diagram, and the Pathway Enrichment Analysis

The main active ingredient of leeches in Chinese medicine is hirudin. Thus, we retrieved a total of 21 compound structures by using the PubChem database (https://https://pubchem.ncbi.nlm.nih.gov//) and subsequently used the CTD database (http://https://ctdbase.org/) to predict the target proteins of hirudin. We constructed the PPI network diagram of the potential target proteins with the STRING database and used the KOBAS 3.0 database for enrichment analysis of the KEGG pathway.

### 2.7. Animal Model Establishment and the Design

We acquired our male SD rats from the Animal Resource Center of Chongqing Medical University (Chongqing, China). The standard diet and free access to water were both given to those rats and kept in cages under a 12 h light/dark cycle. Those male rats with weights of 200 to 250 g were to be utilized in all of the following experiments. All the experiments went along with established principles of the Care and Use of Laboratory Animal in Chongqing Medical University (Chongqing, China).

Following the course of UUO operation, all the rats were anesthetized with 2% pentobarbital sodium salt. A longitudinal incision was made on the left back of rats to expose the left kidney to find the left ureter. The upper part was ligated near the renal pelvis, and the lower part was ligated at the upper third of the ureter. Rats being utilized in the UUO were randomly separated into 2 groups, with 12 rats in one group, which are UUO group (UUO) and an UUO hirudin treatment group (hirudin). Besides, we added an additional sham-operated group (sham) to eliminate the experimental errors from the operation, in which normal rats were given sham operations. After that, rats in the hirudin group were given hirudin (10 IU/kg/d) by tail vein injection and the hirudin was acquired from Canton Xike Kang Biotechnology Co., Ltd., (patent no. ZL03113566.8, 100 IU/vial, Guangxi, China). Correspondingly, both the rats in the sham-operated group and UUO group were given with the normalized saline tail vein injection. Fourteen days after the treatment, before all the rats were sacrificed and the abdominal aortic blood was collected, their kidneys were harvested for histological and biochemical analysis so that we were to estimate hirudin's efficacy in renal fibrosis.

### 2.8. Histopathology

The kidney tissue was collected, and fixation lasted for 24 h in 4% paraformaldehyde to initiate the histological assay. Then tissue was embedded in paraffin and sectioned into 5 *μ*m slices. After the slices were baked for 30 min at 65°C, dewaxing and hydration treatment was conducted. The haematoxylin and eosin (HE) staining and Masson's trichrome staining were used to determine the pathological changes and collagen deposition.

### 2.9. Biochemical Analysis

The creatinine (Scr) content in serum was examined by following the instructions of the Creatinine Assay Kit (Nanjing Jiancheng Bioengineering Institute, China).

### 2.10. Statistical Analysis

The data analysis was conducted by employing SPSS 22.0 software (IBM SPSS Statistics, UAS), and results were expressed as $\bar{x}\pm s$. *T* test was used for the data conforming to normal distribution to determine comparisons between two groups. *P* < 0.05 is thought to be statistically significant.

## 3. Results

### 3.1. Hirudin Inhibits EMT of NRK-52E (Rat Renal Tubular Epithelial Cells)

Through experiments, the efficacy of hirudin on NRK-52E EMT was verified. And the migration ability of the three groups of cells was observed by transwell experiment. We performed WB and qPCR experiments to detect the levels of fibronectin, vimentin, N-cadherin, TGF-*β*, and snail in cells and immunofluorescence to detect the fibronectin and N-cadherin deposition. The results of the transwell experiment are shown in Figure 1(a) indicating that hirudin could significantly inhibit the migration of NRK-52E cells. WB and qPCR experiments showed that the levels of fibronectin, N-cadherin, vimentin, TGF-*β*, and snail in model+hirudin were greatly lower than those in model in which these protein expressions were significantly increased than control (Figures 1(b)–1(d)). The corresponding immunofluorescence results also illustrated that the deposition of fibronectin and N-cadherin in the model+hirudin group was remarkably decreased in contrast to that in model, which confirmed hirudin's ability in inhibiting the EMT of NRK-52E (Figure 2).

### 3.2. PPI Analysis of Hirudin

The CTD database predicted 17 hirudin targets, which were PIK3CG, PIK3CA, AKT, ROS1, TESC, TSC1, TSC2, F2, SERPINE1, MPO, PDGFB, CGB5, CRP, F2R, F2RL3, P2RY12, and SELP (Figure 3(a)). We used the STRING database to construct a PPI network for 17 target proteins (Figure 3(b)) and performed GO analysis and KEGG analysis on these genes (Figures 3(c) and 3(d)). The results expressed that these genes are highly involved in the PI3K/AKT signaling pathway.

### 3.3. Hirudin Reduces the Phosphorylation of PDGFR-*β* and Hinders the Downstream AKT Pathway

This section verified the effect of the combination of hirudin and PDGF on the downstream signaling. WB assay was carried out to verify the efficacy of hirudin on the PDGFB receptor and PI3K/AKT pathway. WB relative quantification results revealed the significant decreasement of p-PDGFR*β*, p-PI3K, and p-AKT protein expression in the model+hirudin group as compared to model (Figure 4). These findings exhibit that hirudin can significantly reduce the phosphorylation level of PDGFR*β* and hinders the PI3K/AKT pathway to achieve the inhibitory efficacy on EMT.

### 3.4. In Vivo Experiments Confirm That Hirudin Reduces Renal Fibrosis in Rats

HE staining micrographs indicated that the UUO group showed severe renal tubule expansion or atrophy, RIF, and inflammatory cell infiltration. Masson staining indicated a large amount of renal interstitial collagen deposition in the UUO group. In contrast, the UUO+hirudin group showed a reversal of the histological changes of the UUO group (Figure 5(a)). The analysis of renal tubular injury score and fibrotic area further confirmed these observations (Figures 5(b) and 5(c)). Compared to sham, the Scr level was significantly elevated in the UUO group, while the hirudin addition group could reduce the Scr level (Figure 5(d)). WB indicated the significant reduction of the marker proteins of RIF in the UUO+hirudin group including fibronectin, collagen III, and *α*-SMA, compared with the UUO group (Figures 5(e) and 5(f)). The above results all verified the significant reduction effect of hirudin on RIF in rats.

### 3.5. In Vivo Experiments Have Verified That Hirudin Reduces EMT in Rats by Repressing the PI3K/AKT Pathway

In this section, we performed WB and qPCR experiments to detect EMT indicators and PI3K/AKT pathways to verify the inhibitory efficacy of hirudin on EMT and PI3K/AKT pathways in rats. The fact that vimentin, N-cadherin, TGF-*β*, and snail are expressed in smaller portion in the UUO+hirudin group in contrast to UUO (Figure 6) suggests that hirudin inhibits the increase of EMT induced by RIF in vivo. Further, we found that the expressions of p-PDGFR*β*, p-PI3K, and p-AKT in the UUO+hirudin group were markedly relieved (Figure 7) when compared with the UUO group, confirming the inhibitory efficacy of hirudin on EMT by repressing the PI3K/AKT pathway in vivo. These results were consistent with those of in vitro cell experiments.

## 4. Discussion

Obesity, diabetes, hypertension, and increased human life span are all causes of CKD. RIF is the final pathological manifestation of most CKD patients and a precursor of end-stage renal disease [20]. RIF is a pathological phenomenon, mainly manifested by the deposition of ECM and the activation and proliferation of fibroblasts [21]. Recent studies have found that the renal tubular EMT is one of the important pathogenesis of RIF, but the pathogenesis of RIF is very complicated [22]. Therefore, renal tubular EMT has not only become a breakthrough in the treatment of chronic kidney disease but has also gradually become a research hotspot. Tubular EMT implies the transformation of renal tubular epithelial cells into fibroblasts or myofibroblasts [23]. The intuitive manifestations at the molecular level are decreased expression of cell epithelial markers such as E-cadherin, cytokeratin, and tight junction protein-1, accompanied by increased deposition of intercellular markers including vimentin, *α*-SMA, and fibroblast-specific proteins, leading to a result of cells gaining the ability to migrate into the interstitial and ECM synthesis increasing [24–26].

With the increasing incidence of kidney diseases in recent years, there are more and more reports about hirudin in the treatment of kidney diseases. Some research teams injected the recombinant hirudin/liposome complex into a rat model of nephropathy and found that that complex promoted the deposition of hirudin in the renal tissue and reduced kidney damage in the rat [27]. The codeposition of IgA and IgG is considered as the features of immunoglobulin A nephropathy (IgAN). Studies have found that in the IgAN model, hirudin improved the accumulation of apoptosis-associated proteins (Caspase3 and Caspase9) by decreasing serum creatinine, proteinuria, and urea nitrogen levels, thereby repressing fibrosis and inflammation to achieve the purpose of improving IgAN [28]. Robson et al. believed that the pharmacokinetics of hirudin is linearly related, dose-dependent, and independent of gender; the metabolism of hirudin in the body is completed by the kidneys: about 20% of the drug is eliminated by the kidneys, which supplies a blood concentration foundation for the application of hirudin in the treatment of kidney diseases [29]. At present, research reports have made it clear that hirudin can reduce RIF by modulating the NF-*κ*B and TGF-*β*1/Smad pathway, but there is no correlated publication on the efficacy of hirudin on EMT and RIF [18]. This study first confirmed the inhibitory effect of hirudin on EMT of renal tubular epithelial cells and revealed the role of hirudin in reducing the phosphorylation level of PDGFR*β*, thereby inhibiting the PI3K/AKT signaling.

Firstly, we estimated the inhibitory efficacy of hirudin on EMT of NRK-52E cells. On the basis of the results of transwell, we found that the model+hirudin group has a significantly lower cell number than the model group, suggesting that hirudin dramatically inhibits the migration ability of renal tubular epithelial cells.Secondly, through protein and mRNA level determination experiments to detect EMT indicators such as fibronectin, N-cadherin, vimentin, TGF-*β*, and snail, the results revealed that hirudin markedly inhibited the expressions of EMT indicators. In addition, we also did the immunofluorescence of N-cadherin and vimentin and got the same conclusion. Finally, we explained the inhibitory efficacy of hirudin on EMT of NRK-52E cells: with the help of the CTD database, 17 target proteins of hirudin were obtained. PDGF is a peptide regulator discovered in 1974 to stimulate tissue cell growth, and it exists in platelet granules in physiological state and is activated and released by disintegrating platelets when blood coagulation and has biological activity to stimulate chemotactic and growth of specific cells. The PDGF family consists of 4 PDGF genes, namely, PDGFA, PDGFB, PDGFC, and PDGFD. These genes are located on human chromosomes 7, 22, 4, and 11 and mouse chromosomes, 15, 3, and 9, respectively. There are 5 bioactive proteins in the PDGF family. In addition to 4 homologous dimers (PDGF-AA, PDGF-BB, PDGF-CC, and PDGF-DD), there is also a heterodimer, PDGF-AB [30]. The PDGF family is a key factor in the normal development of embryos, cell growth and differentiation, and response to tissue damage. Many pathological processes are related to the abnormal activity of PDGF and its receptors. PDGFR serves as a crucial member in tyrosine protein kinase family and is capable of promoting cell differentiation, proliferation, invasion, and migration [30].

Further, KOBAS 3.0 was used for KEGG pathway enrichment analysis of 17 target proteins of hirudin. These protein molecules are mainly enriched in complement and coagulation cascade, platelet activation, Rap1 signaling, neuroactive ligand-receptor interaction, modulation of actin cytoskeleton, cancer pathway, phospholipase D signaling, PI3K/AKT signaling pathway, etc. PI3K/AKT is a typical signaling pathway that modulates cell growth, metastasis, apoptosis, and drug resistance. In recent years, reports have demonstrated the regulatory effect of the PI3K/AKT pathway in EMT. EMT activation requires cytokine participation like PDGF, TNF-*α*, and TGF-*β* [5, 31]. The combination of the p85 unit of PI3K with phosphorylated PDGFR first activates the downstream molecule serine/threonine kinase and further leads to the final activation of AKT [13].

Finally, we also answered the fact that hirudin has an effect on the PI3K-AKT pathway. Through WB and qPCR, we confirmed that hirudin can downregulate the activation of the PI3K/AKT pathway caused by EMT in NRK-52E. In addition, we also found that hirudin reduced the phosphorylation level of PDGFR*β*, which suggests that the molecular mechanism of hirudin in inhibition of rat renal tubular epithelial cells is most likely to inhibit the PI3K/AKT pathway by reducing the phosphorylation level of PDGFR*β*. UUO operation is a typical model of renal tubule fibrosis, which is characterized by renal interstitial inflammation, extracellular matrix deposition, tubule expansion, atrophy, and fibrosis. Its molecular mechanism is extremely complex and includes the involvement of inflammatory mediators, fibrogenic factors, oxidative stress, and apoptosis [16, 32]. After the UUO model was constructed, we also confirmed that hirudin significantly reduced the level of renal interstitial fibrosis, severe tubular dilatation or atrophy, inflammatory cell infiltration, and massive accumulation of interstitial collagen in the model group in rats. The decreased EMT relevant molecules and PI3K-AKT signaling pathway proteins were confirmed by WB and qPCR in UUO rats after hirudin treatment. At the same time, we also confirmed that hirudin also inhibits EMT caused by PI3K-AKT by reducing the phosphorylation of PDGFR*β* in vivo.

## 5. Conclusion

We found that the molecular mechanism of hirudin in renal fibrosis treatment may be that hirudin inhibits the PI3K/AKT signal pathway by reducing the phosphorylation level of PDGFR*β*. This investigation is predicted to bring about a theoretical foundation for the clinical application of hirudin in treating chronic kidney disease and in reversing renal interstitial fibrosis and contribute to proposing a potential target of hirudin.

## Figures and Tables

**Figure 1:** Hirudin's inhibition towards the EMT indicators of NRK-52E. (a) The cell migration conditions of the control, model, and hirudin group are revealed by transwell assay. Scale bar: 100 *μ*m. (b) The western blot assay on the protein expressions of fibronectin, N-cadherin, vimentin, TGF-*β*, and snail and (c) the corresponding gray statistics parameters. (d) The qPCR detection on the expressions of fibronectin, N-cadherin, vimentin, TGF-*β*, and snail. ^##^*P* < 0.01, compared with the model.

**Figure 2:** Hirudin's inhibition towards the EMT of NRK-52E (rat renal tubular epithelial cells). (a) The protein expression conditions of fibronectin in 3 different groups revealed by immunofluorescence assay. (b) The protein expression conditions of N-cadherin in 3 different groups revealed by immunofluorescence assay. Scale bar: 50 *μ*m. (c) The outcomes of average fluorescence intensity statistical parameters on fibronectin and N-cadherin proteins. ^##^compared with model, *P* < 0.01.

**Figure 3:** Target point analysis outcomes on hirudin. (a) Diagram of hirudin-to-target-protein interactions. (b) PPI analysis on the target proteins. (c) GO analysis. (d) KEGG analysis.

**Figure 4:** Hirudin works out an inhibitory effect on both the overall phosphorylation of PDGFR*β* and the downstream AKT pathway. (a) Western blot detection on the expressions of PDGFB, PDGFR*β*, p-PDGFR*β*, PI3K, p-PI3K, AKT, and p-AKT. (b) Semiquantitative analysis was performed based on the gray value. GAPDH was used for the endogenous protein. ^##^compared with the Model, *P* < 0.01.

**Figure 5:** Alleviating ability of hirudin on the renal fibrosis of rat. (a) HE staining and Masson staining. Scale bar: 50 *μ*m. (b) Scoring on renal tubule injury condition. (c) Fibrotic area on fibrosis condition. (d) Evaluation on Scr content. (e) Western blot detection to reveal the expressions of fibronectin, collagen III, and *α*-SMA. (f) Semiquantitative analysis was performed based on the gray value. GAPDH was used for the endogenous protein. ^##^compared with UUO, *P* < 0.01.

**Figure 6:** Detection on the expressions of the EMT relevant molecules. (a) The western blot assay to reveal the expressions of N-cadherin, vimentin, TGF-*β*, and snail. (b) Semiquantitative analysis was performed based on the gray value. GAPDH was used for the endogenous protein. (c) The qPCR detection on the expressions of N-cadherin, vimentin, TGF-*β*, and snail. ^##^compared with UUO, *P* < 0.01.

**Figure 7:** Detection on the expressions of the PI3K/AKT pathway. (a) The western blot assay to reveal the expressions of PDGFB, PDGFR*β*, p-PDGFR *β*, PI3K, p-PI3K, AKT, and p-AKT. (b) Semiquantitative analysis was performed based on the gray value. GAPDH was used for the endogenous protein. ^##^compared with UUO, *P* < 0.01.

## Data Availability

The data used to support the findings of this study are included within the article.
